The article "Extensive Pulmonary Embolism Following Mild COVID-19 Pneumonia" was retracted in 2024. Reasons: false authorship; unreliable results or conclusions; no approval from an author; concerns about the authorship.

# Extensive Pulmonary Embolism Following Mild COVID-19 Pneumonia

**DOI:** 10.7759/cureus.21436

**Published:** 2022-01-19

**Authors:** Ruba M Barnawi, Turki A Alsulami, Waleed A Alzahrani, Abdullah M Alsharif, Mohammed A Alsalaim, Ziyad A Alqazlan, Mohammed A Aljawi, Abdulaziz H Alghamdi, Mohammed A Alzubaidi, Zainab A Alqaysum, Hasan A Alabbad, Zied A Aljubour, Gadeer A Albannawi, Maryam M Alfaqih, Faisal Al-Hawaj

**Affiliations:** 1 Medicine, King Saud University, Riyadh, SAU; 2 Medicine, Debrecen University, Debrecen, HUN; 3 Medicine, Taif University, Taif, SAU; 4 Medicine, Almmarefa University, Riyadh, SAU; 5 Medicine, Najran University, Najran, SAU; 6 Medicine, Qassim University, Qassim, SAU; 7 Medicine, Taif Universty, Taif, SAU; 8 Medicine, Ibn Sina National College for Medical Studies, Jeddah, SAU; 9 Medicine, Jordan University of Science and Technology, Irbid, JOR; 10 Medicine, Imam Abdulrahman Bin Faisal University, Dammam, SAU; 11 Medicine, King Faisal Uneversity, Hofuf, SAU; 12 Medicine, Almareefa University, Riyadh, SAU; 13 Medicine, Umm Al-Qura University, Mecca, SAU

**Keywords:** case report, inferior vena cava thrombosis, pulmonary embolism, coagulopathy, covid-19, thrombosis

## Abstract

The coronavirus disease 2019 (COVID-19) is caused by the severe acute respiratory syndrome coronavirus 2 (SARS-CoV-2) and predominantly manifests with respiratory symptoms. However, it may have a wide range of complications, including hematological complications. Several studies demonstrated that patients with COVID-19 exhibit a wide range of complex abnormalities of the coagulation system. We report the case of a 22-year-old man who presented to our emergency department with a cough and fever for one week. His vital signs were normal. Since the patient was young and mildly symptomatic, he was offered the option of home isolation for seven days. Two weeks later, the patient presented to the emergency department complaining of sudden shortness of breath that was associated with chest pain. The oxygen saturation was 92% on room air. The patient underwent computed tomography pulmonary angiography. The scan showed a centric filling defect in the main right and left pulmonary arteries representing pulmonary embolism. Further, the scan showed a thrombus in the inferior vena cava that was the source of bilateral pulmonary embolism. The patient was admitted to the intensive care unit. He received full anticoagulation with heparin. After recovery, he underwent a thrombophilia screen, which yielded normal findings. The present case demonstrated that thromboembolic events may develop even after the recovery from mild COVID-19 pneumonia. In the appropriate clinical settings, physicians should maintain a high index of suspicion of coagulopathy in any patient with recent COVID-19 pneumonia. Further studies are needed to determine the indication and duration of the thromboprophylaxis following the recovery from COVID-19.

The article "Extensive Pulmonary Embolism Following Mild COVID-19 Pneumonia" was retracted in 2024. Reasons: false authorship; unreliable results or conclusions; no approval from an author; concerns about the authorship.

## Introduction

The coronavirus disease 2019 (COVID-19) is caused by the severe acute respiratory syndrome coronavirus 2 (SARS-CoV-2) and predominantly manifests with respiratory symptoms. However, COVID-19 can be considered a multi-organ disease. It may have a wide range of complications, including gastrointestinal, hepatobiliary, neurological, and hematological complications. Several studies demonstrated that patients with COVID-19 exhibit a wide range of complex abnormalities of the coagulation system [1,2]. The coagulopathy resulting from COVID-19 can be explained by Virchow’s triad that includes endothelial injury, stasis, and hypercoagulable states. It has been shown that the SARS-CoV-2 may directly invade the endothelial cells, which can lead to the initiation of the coagulation pathway. Further, immobilization in hospitalized patients is an independent risk factor for thrombosis [3]. Additionally, it is reported that several prothrombotic factors are to be increased in patients with COVID-19, including factor VIII and fibrinogen. Further, there is a growing body of evidence that thrombotic complications may develop even after discharge from COVID-19 [4]. Here, we report the case of a previously healthy young adult with extensive pulmonary embolism developing following the recovery from mild COVID-19 pneumonia.

## Case presentation

A 22-year-old man presented to our emergency department with a cough and fever for one week. The cough was not productive of sputum. The fever was intermittent and its maximum measurement was 38.1℃ and showed complete resolution with paracetamol. Five days before his symptoms, he had contact with his friend who was later tested positive for SARS-CoV-2. The patient was healthy with no remarkable comorbidity. He maintained an active lifestyle. He had no history of smoking, alcohol, or recreational drug use. Physical examination, including vital signs, showed no abnormalities. The polymerase chain reaction testing for SARS-CoV-2 yielded positive results. Since the patient was young and mildly symptomatic, he was offered the option of home isolation for seven days.

Two weeks later, the patient presented to the emergency department complaining of sudden shortness of breath that was associated with chest pain. There was no history of cough or wheezing. His vital signs showed tachycardia (130 bpm), tachypnea (25 bpm), and maintained blood pressure. The oxygen saturation was 92% on room air. The initial laboratory investigation, including leukocytes and C-reactive protein, was normal. However, the D-dimer level was elevated (1.3 g/L). Further, a portable chest radiograph was performed and showed clear lung fields (Figure 1).

The article "Extensive Pulmonary Embolism Following Mild COVID-19 Pneumonia" was retracted in 2024. Reasons: false authorship; unreliable results or conclusions; no approval from an author; concerns about the authorship.

**Figure 1:** Frontal chest radiograph shows clear lung fields with no infiltrates.

In order to rule out pulmonary embolism as the causative etiology of decreased oxygen saturation, the patient underwent computed tomography pulmonary angiography. The scan showed a centric filling defect in the main right and left pulmonary arteries representing pulmonary embolism (Figure 2). Further, the interventricular septum appears straightened suggesting the presence of right ventricular strain.

**Figure 2:** CT pulmonary angiography shows bilateral pulmonary embolism (arrows). CT: computed tomography

Subsequently, the patient underwent bilateral duplex venous ultrasound examination. It revealed that the common femoral, superficial femoral, and popliteal veins have normal lumen with normal compressibility and normal color flow. Abdominal angiography was performed to identify any possible location of the primary thrombus. The computed tomography revealed that there was a thrombus in the inferior vena cava that was the source of bilateral pulmonary embolisms (Figure 3).

**Figure 3:** CT abdominal angiography shows a filling defect (arrow) in the inferior vena cava representing a thrombus. CT: computed tomography

The patient was admitted to the intensive care unit. He received full anticoagulation with unfractionated heparin. His condition showed gradual improvement. He did not require inotrope or mechanical ventilation support during his stay. After eight days, he was discharged with close regular follow-up. Then, he underwent a thrombophilia screen, which yielded normal findings.

## Discussion

We reported the case of an extensive pulmonary embolism following the recovery from COVID-19 pneumonia. Several clinical lessons can be drawn from this case report. The case demonstrated the coagulopathy may persist even after the recovery from COVID-19 pneumonia. Further, coagulopathy complications may occur even in patients with mild respiratory disease that can be managed with home isolation.

Coagulopathy in COVID-19 has a wide spectrum of clinical presentations with variable severity ranging from asymptomatic to organ dysfunction and death. From the early period of COVID-19, it has been recognized that venous thromboembolic diseases, including deep venous thrombosis and pulmonary embolism, are very prevalent among acutely ill patients [5]. Further, the coagulopathy complications may include arterial events resulting in a stroke, myocardial infarction, and limb ischemia [6]. Further, microvascular thrombosis has been described in postmortem examination for patients with COVID-19 pneumonia [7].

The article "Extensive Pulmonary Embolism Following Mild COVID-19 Pneumonia" was retracted in 2024. Reasons: false authorship; unreliable results or conclusions; no approval from an author; concerns about the authorship.

The present case is consistent with the available literature that showed an increased risk of venous thrombosis following the recovery from COVID-19 pneumonia. For example, Patell et al. [4] found that up to 2.5% of 19 patients developed a thromboembolic event within 30 days of discharge from COVID-19 pneumonia. They concluded that there is a pressing need to investigate the role of thromboprophylaxis after the discharge from COVID-19.

A recent randomized controlled trial, involving 320 patients, investigated the benefit of the use of rivaroxaban as a thromboprophylaxis after the recovery from COVID-19 and showed that patients in the treatment group developed a significantly lower number of venous thrombosis events compared with the control group with no higher incidence of major bleeding complications [8]. However, it seems unlikely that clinicians will adhere to the recommendation of thromboprophylaxis after COVID-19 until more evidence become available.

## Conclusions

The present case demonstrated that thromboembolic events may develop even after the recovery from mild COVID-19 pneumonia. In the appropriate clinical settings, physicians should maintain a high index of suspicion of coagulopathy in any patient with recent COVID-19 pneumonia. The case suggested that thromboprophylaxis might be recommended in a selected group of patients after the recovery from COVID-19 pneumonia. However, further studies are needed to determine the indication and duration of the thromboprophylaxis following the recovery from COVID-19.
